The article "MEA-CNDP: A Membrane Evolutionary Algorithm for Solving Biobjective Critical Node Detection Problem" was published in 2021. Journal: Comput Intell Neurosci.

# MEA-CNDP: A Membrane Evolutionary Algorithm for Solving Biobjective Critical Node Detection Problem

**DOI:** 10.1155/2021/8406864

**Published:** 2021-11-28

**Authors:** Yaochang Xu, Ping Guo

**Affiliations:** ^1^College of Computer Science, Chongqing University, Chongqing 400044, China; ^2^Chongqing Key Laboratory of Software Theory and Technology, Chongqing 400044, China

## Abstract

The critical node detection problem (CNDP) refers to the identification of one or more nodes that have a significant impact on the entire complex network according to the importance of each node in a complex network. Most methods consider the CNDP as a single-objective optimization problem, which requires more prior knowledge to a certain extent. This paper proposes a membrane evolution algorithm MEA-CNDP to solve biobjective CNDP. MEA-CNDP includes a population initialization strategy based on the evaluation of decision variables, a strategy to transform the main objective, a strategy to update the membrane inherited pool, and four membrane evolutionary operators. The numerical experiments on 16 benchmark problems with random and logarithmic weights show that MEA-CNDP outperforms other algorithms in most cases. In particular, MEA-CNDP has unique advantages in dealing with large-scale sparse bi-CNDP.

## 1. Introduction

The nature-inspired optimization strategy has shown very interesting results in many fields, such as teach optimization techniques and so on [1]. As a new branch of natural computing, membrane computing has attracted continuous attention of researchers, it is a computing model abstracted from biological cells, organs, and tissues. Based on the cell membrane, the membrane computing establishes a calculation model based on the function and characteristics of the cell membrane. Such a calculator is also called the P system. Membrane computing has been widely concerned since it was proposed, and it has shown excellent results in many applications. Most P systems have been proved to have the same computing power as Turing machines [2, 3]. In theory, many NP-hard problems can also be solved in polynomial time using the P system, such as the all-set problem [4] and Hamilton loop problem [5]. Since membrane computing was put forward, it has received extensive attention and has been applied in many fields, such as image processing [6], numerical optimization [7], and social network analysis [8].

Inspired by membrane computing, Nishida combined membrane nested structure with other evolutionary algorithms in 2004 and proposed the membrane algorithm framework (MA) for the first time [9]. Since then, researchers call the algorithms based on this framework membrane algorithm, which provides a nested structure compatible with other algorithms, making MA well combined with various algorithms to solve different problems. For example, a membrane clustering algorithm for automatic clustering is proposed in [10] based on MA, which can easily find the number of clustering under the control of evolutionary communication mechanism. Combining particle swarm optimization (PSO) and MA, a membrane heuristic algorithm based on particle swarm optimization (mMPSO) is proposed to solve the path planning problem of multiobjective robots in dynamic obstacles and dangerous environments [11]. Moreover, in [12], MA is combined with differential evolution algorithm (DE), in [13], and MA is combined with quantum evolution algorithm (QEA).

The article "MEA-CNDP: A Membrane Evolutionary Algorithm for Solving Biobjective Critical Node Detection Problem" was published in 2021. Journal: Comput Intell Neurosci.

Based on MA, membrane evolutionary algorithm (MEA) is introduced, MEA is an evolutionary algorithm framework inspired by the behavior characteristics of biological cells. It simulates various life activities of cells, realizes information exchange between cells by relying on membrane, and thus realizes individual evolution. In [14], a membrane evolutionary algorithm for solving minimum vertex cover problem (MEAMVC) is introduced, and the experimental results show that the MEAMVC has good performance in solving the minimum vertex coverage problem. In [15, 16], MEA are introduced to solving the maximum clique problem and travelling salesman problem, respectively.

A crucial research direction in engineering design is to consider optimization problems. With the continuous increase of the scale of optimization problems and the increase of dynamic and random factors, traditional methods reflect the complexity and instability of calculation. Therefore, researchers are looking for various new methods to solve optimization problems. In recent years, some excellent methods have emerged and have been applied to various fields. For example, Zapata et al. [17] propose that a novel hybrid swarm algorithm combining strengths of self-assembly and the particle swarm optimization greatly improves the convergence speed. Reference [18] presents a novel application of the metaheuristic slime mould algorithm (SMA) to the optimal tuning of interval type-2 fuzzy controllers. Population-based evolutionary algorithm has shown gratifying results in solving optimization problems, and a new estimation of distribution algorithm (EDA) is introduced in [19]. It maintains a trade-off between run time and the number of evaluation points. Reference [20] combines the island model and cuckoo search (CS) algorithm and thus presents the island-based CS with polynomial mutation (iCSPM), which greatly improves the search ability and maintains the population diversity.

The article "MEA-CNDP: A Membrane Evolutionary Algorithm for Solving Biobjective Critical Node Detection Problem" was published in 2021. Journal: Comput Intell Neurosci.

Complex networks can be seen everywhere in both scientific research and daily life. As an important subject of optimization problems, the critical node detection problem (CNDP) aims to identify the critical nodes in complex networks, which is also a common means to study graph problems. Similar problems include the critical node problem (CNP), which aims to minimize the connectivity of the residual graph under the constraint of the maximum number of nodes that can be deleted [21]. Cardinality-constrained critical node detection problem (CC-CNP) is devoted to minimizing the number of deleted nodes given the maximum connected component [22].

At present, the methods to solve CNDP mainly include accurate algorithm and heuristic algorithm. For the accuracy strategy, most algorithms consider CNDP as an integer programming problem [23–25], which has significant limitations. In contrast, the heuristic algorithm has achieved good results in solving CNDP. A hybrid heuristic algorithm is proposed with the combination of greedy algorithm and local search algorithm and shows good performance in [26]. In [27], incremental learning based on population is combined with a simulated annealing optimization algorithm based on combinatorial rank free problem representation to solve CNDP, which saves space and reduces the need for individual repair mechanism simultaneously.

Most of the above algorithms treat CNDP as a single-objective optimization problem. Among them, the maximum number of nodes that can be deleted and the maximum number of connected components are often required. However, in practical problems, prior knowledge is often not easy to obtain. Moreover, considering the network connectivity and the cost of deleting nodes are often two conflicting objectives, which should be viewed simultaneously. Therefore, establishing a biobjective optimization model for CNDP is considerable. In [28], CNDP is considered a biobjective optimization problem for the first time, and the Pareto fronts of some problems are given. In [29], a specific biobjective optimization model of CNDP is proposed, and the ant colony algorithm is used to solve it. In [30], a biobjective optimization model for CNDP is established, and the two objective functions are the number of connected components and their cardinal variance, respectively, but this is actually a generalization of pairwise connectivity.

This paper proposes a novel evolutionary algorithm based on MA for solving the biobjective critical node detection problem (bi-CNDP) model in [31], called MEA-CNDP for short. Based on membrane division, differentiation, death, and other life activities, MEA-CNDP designs and implements four evolutionary operators: division, fusion, cytolysis, and selection operator. Aiming at bi-CNDP, a new population initialization strategy is proposed in MEA-CNDP, and the main objective transforming and membrane-to-subproblem matching strategy are adopted to improve the efficiency of MEA-CNDP. The main contributions of this paper include the following:

- Taking into account the characteristics of bi-CNDP, a new population initialization strategy based on the evaluation of decision variables is proposed. By calculating the number of nondominated front and the cost of nodes, the importance of each decision variable can be levelled out, thereby generating a high-quality initial population.
- Design and implement four evolutionary operators, including division, fusion, cytolysis, and selection operator. By the communication between membranes, those evolutionary operators can generate better individual membrane, eliminate the membrane with poor quality, and update the external archive membrane.
- A membrane evolutionary algorithm MEA-CNDP is proposed to solve the bi-CNDP. The experimental results on four different types of instances show that the MEA-CNDP algorithm has unique advantages in dealing with large-scale sparse bi-CNDP.

The article "MEA-CNDP: A Membrane Evolutionary Algorithm for Solving Biobjective Critical Node Detection Problem" was published in 2021. Journal: Comput Intell Neurosci.

The rest of this paper is organized as follows.  Section 2 introduces the basic knowledge and related definition, including the concept of MA and MEA, CNDP, and bi-CNDP. Moreover, some algorithms solving bi-CNDP are introduced briefly. In Section 3, the framework of MEA-CNDP is proposed, and the details of related strategies for improving the efficiency are introduced; at last, the implementation of four types of evolutionary operators is detailed. In Section 4, based on four types of bi-CNDP instances, the comparative experiments are designed, and the analysis of the experimental results is given as well, which verified the performance of MEA-CNDP. Finally, the conclusion and future work are drawn in Section 5.

## 2. Preliminaries

This section provides the related research basis of this paper. Firstly, the related content of membrane computing is introduced, and the related knowledge of MEA is submitted. Then, the related definition and formula of CNDP are presented briefly, thus providing the multiobjective optimization problem (MOP) model of CNDP, that is, the biobjective critical node detection problem (denoted as bi-CNDP). Finally, some related algorithms solving bi-CNDP are introduced briefly, which are used in the subsequent comparative experiments.

### 2.1. Membrane Algorithm and Membrane Evolutionary Algorithm

As a biological computing model abstracted from the level of biological cells, membrane computing is committed to studying the function and characteristics of the cell membrane in organisms and applying them to optimization problems; such a calculator is also called a P system [32]. P system is mainly composed of its structure, material object, and evolutionary rules. The main body of the P system is to construct the membrane structure corresponding to specific problems by simulating the basic structure of the cell membrane. Evolutionary rules are the basis of material communication within and between membranes. Different rules are implemented to transform different information.

The article "MEA-CNDP: A Membrane Evolutionary Algorithm for Solving Biobjective Critical Node Detection Problem" was published in 2021. Journal: Comput Intell Neurosci.

MA is an algorithm framework derived from membrane computing. MA provides a nested structure compatible with various other algorithms, enabling various excellent algorithms to solve the final problem in the framework of membrane computing, aiming at specific subproblems, giving full play to their respective advantages.

The nested structure of MA is shown in Figure 1. The main structural feature of MA is a layer of nested membranes. The region between each two nested membranes contains subalgorithms. In different regions, the subalgorithms can be the same or different. These subalgorithms usually solve different stages of the problem or solve different parts of the problem.

MEA is an evolutionary algorithm based on cell division, fusion, death, and other life activities, according to the characteristics of the cell membrane to achieve information exchange between cells. According to the life activities of cells and the information exchange mechanism between cells, MEA designs the operators of division, fusion, cytolysis, and selection and uses the membrane parallel optimization and heuristic information to realize individual evolution and further solve the problem.

The algorithm framework of the membrane evolutionary algorithm is shown in Algorithm 1. The framework of MEA includes four parts: population and membrane structure initialization, membrane evolution, membrane repair, and final solution output.

The primary evolutionary process of MEA is the four operators of division, fusion, cytolysis, and selection. The membrane population is constantly operating these four operators to make the whole population evolve in a better direction.

- Division operator: in MEA, one individual membrane divides into two submembranes, the substance in the original individual membrane is distributed into the two submembranes, and the original individual membrane is removed. The process of division operator is shown in Figure 2(a).
- Fusion operator: in MEA, the fusion operator merges two individual membranes into one membrane, and all the substances in the original two membranes enter into the newly formed membrane, while the original two membranes and their substances are removed. The process of the fusion operator is shown in Figure 2(b).
- Cytolysis operator: in MEA, the individual membrane with poor performance or without specific conditions will be dissolved, and the dissolved substances in the membrane can be deleted or released into the environmental membrane.
- Selection operator: in MEA, the membrane with higher fitness or better individuals should be retained, and the selection operator is used to update the excellent individuals in the membrane population evolution.

The article "MEA-CNDP: A Membrane Evolutionary Algorithm for Solving Biobjective Critical Node Detection Problem" was published in 2021. Journal: Comput Intell Neurosci.

In MEA, each individual membrane is regarded as a candidate solution, and information exchange and synchronization are realized among multiple individual membranes; thus, the whole membrane population evolves in a better direction. Precisely because of such characteristics, MEA possesses remarkable parallelism and scalability, flexible coding, and excellent search capability.

### 2.2. CNDP and Bi-CNDP

CNDP refers to the identification of one or more nodes that can significantly affect the entire complex network based on the different importance of each node in the complex network. The significant impact here includes the promotion or mitigation of the entire complex network.

Let *G*=(*V*, *E*) be an undirected weighted graph, the number of nodes is |*V*|=*n*, and the number of edges is |*E*|=*m*. The goal of CNDP is to determine a subset *R*⊆*V*, so that the residual graph *G*(*V*\*R*) has the minimum number pairwise connectivity (i.e., the number of a pair of nodes connected by a path in a graph), where |*R*| ≤ *K*, *K* is the maximum number of the deleted nodes allowed. If the nodes of CNDP are weighted, that is, the weighted critical node detection problem (denoted as wCNDP) transforms the constraint to *ω*_*R*_ ≤ *ω*, where the *ω*_*R*_ is the sum of the weights of the deleted nodes and *ω* is the maximum weights of the deleted nodes allowed. More detailed about wCNDP can be seen in [30].

To solve the CNDP as a single-objective optimization problem, it is often required to give the maximum number of deleted points or determine the maximum number of connected components. However, in practical issues, the prior knowledge is often not easy to obtain, and considering the network connectivity and the cost of deleted nodes are often two conflicting objectives, which should be viewed simultaneously. Therefore, it is of great value to establish a biobjective optimization model for CNDP.

The model of bi-CNDP is introduced in [31], which considers the pairwise connectivity and the cost of deleting nodes simultaneously. Let *G*=(*V*, *E*, *C*) be a weighted undirected graph, *V*={*v*_1_, *v*_2_,…, *v*_*n*_} is the set of nodes of *G*, *E*={(*v*_*i*_, *v*_*j*_)*|i*, *j* ∈ {1,2,…, *n*}} is the set of edges, and the cost of deleting each node is given in *C*={*c*_1_, *c*_2_,…, *c*_*n*_}.

The article "MEA-CNDP: A Membrane Evolutionary Algorithm for Solving Biobjective Critical Node Detection Problem" was published in 2021. Journal: Comput Intell Neurosci.

The first objective function of bi-CNDP is about pairwise connectivity, which can be calculated by

(1) $$\begin{array}{c} \text{PWC}\left(G\right)=\frac{1}{2}\sum_{v_{i},v_{j}\in V,v_{i}\neq v_{j}}x_{ij}, \end{array}$$

where *x*_*ij*_=1 if *v*_*i*_ and *v*_*j*_ are connected; otherwise, *x*_*ij*_=0; it can be further normalized as

(2) $$\begin{array}{c} \text{nPWC}\left(G\right)=\frac{1}{n\left(n-1\right)}\sum_{v_{i},v_{j}\in V,v_{i}\neq v_{j}}x_{ij}, \end{array}$$

It can be seen that the value range of nPWC(*G*) is [0, 1], obviously, nPWC(*G*) can be considered the measure of connectivity of the graph because nPWC(*G*) is proportional to the number of nodes connected through at least one path. The closer the nPWC(*G*) value is to 1, the closer the graph is to the connected graph.

After deleting nodes, except for minimizing the connectivity of the network, minimizing the cost of deleting these nodes is considerable. Therefore, the second objective function of bi-CNDP is used to measure the cost of deleting the selected nodes *R*⊆*V*, which can be calculated by

(3) $$\begin{array}{c} \text{nCost}\left(R\right)=\frac{\sum_{v_{i}\in R}c_{i}}{\sum_{v_{i}\in G}c_{i}}, \end{array}$$

where *c*_*i*_ is the weight associated with *v*_*i*_, ∑_*v*_*i*_∈*G*_*c*_*i*_ is drawn to normalizing, which makes the value range in [0, 1] as well.

Therefore, the model of bi-CNDP can be described as

(4) $$\begin{array}{c} \text{minimize}\left(\text{nPWC}\left(G\left(V\backslash R\right)\right),\text{nCost}\left(R\right)\right),\\ \text{s.t}.\left\{\begin{array}{cc} x_{ij}+y_{i}+y_{j}\geq 1, & \;\forall v_{i},v_{j}\in V,\\ x_{ij}+x_{jk}+x_{ki}\neq 2, & \forall v_{i},v_{j,}v_{k}\in V,\\ x_{ij}\in \left\{0,1\right\}, & y_{i}\in \left\{0,1\right\},\;\forall v_{i},v_{j}\in V, \end{array}\right. \end{array}$$

where *y*=(*y*_1_, *y*_2_,…, *y*_*n*_) is the decision variables, *y*_*i*_ is the binary variable, *y*_*i*_=1 if the node *v*_*i*_ is deleted, and *y*_*i*_=0 otherwise. *x*_*ij*_ shows the connectivity of *v*_*i*_ and *v*_*j*_, *x*_*ij*_=1 if *v*_*i*_ and *v*_*j*_ belong to the same connected component, and *x*_*ij*_=0 otherwise.

*y*=(*y*_1_, *y*_2_,…, *y*_*n*_) is the decision variables to be optimize, *y*_*i*_ values in {0, 1} and changes continuously with the implementation of the programme, until it evolves into a good enough solution. The first constraint ensures that the residual graph after deleting some nodes includes several connected components. The second constraint ensures that, for three nodes in the same connected component, any two nodes between them are also in the same connected component. The third constraint specifies the range of values for *x*_*ij*_ and *y*_*i*_.

The article "MEA-CNDP: A Membrane Evolutionary Algorithm for Solving Biobjective Critical Node Detection Problem" was published in 2021. Journal: Comput Intell Neurosci.

It can be seen that bi-CNDP defined above is NP-hard on the general graph. Although the Pareto front of the above model cannot be obtained for the time being for the general graph, for the CNDP whose graph structure is a tree, the algorithm with polynomial time can get the approximate Pareto front of the above model. Therefore, a heuristic algorithm is needed for general graphs to find the approximate Pareto front of the above bi-CNDP.

### 2.3. Related Algorithms

#### 2.3.1. MOEA/D

The strategy based on decomposition is a practical approach and widely used method in multiobjective optimization evolutionary algorithm, such as the multiobjective evolutionary algorithm based on decomposition (MOEA/D) is proposed in [33]. MOEA/D decomposes the MOP into several scalar single-objective optimization subproblems and then optimizes the subproblems simultaneously. In MOEA/D, each subproblem is optimized only according to the information of its adjacent subproblems, which significantly reduces the computational complexity of each generation.

In MOEA/D, it is crucial to decompose the MOP into multiple scalar subproblems, and the common aggregation functions mainly include the weighted sum approach, Chebychev approach, and boundary intersection approach [34]. MOEA/D firstly introduces the decomposition method into MOP, making the idea of decomposition into the evolutionary algorithm. In addition, by decomposing the MOP into multiple scalar optimization subproblems for optimization, MOEA/D significantly reduces the difficulty of maintaining population diversity and fitness allocation.

#### 2.3.2. DMOEA-*ε*C

Based on MOEA/D, the decomposition-based multiobjective evolutionary algorithm with the *ε*-constraint framework (DMOEA-*ε*C) is proposed in [35]. DMOEA-*ε*C uses the *ε*-constraint method to MOPs, it selects one objective function as the main objective, transforms other objectives into constraints, allocates upper bound vectors for each subproblem, and then optimizes multiple subproblems simultaneously for MOP; the *ε*-constraint formula can be defined as

(5) $$\begin{array}{c} \text{minimize }f_{\text{main}}=f_{s}\left(x\right)+\rho \sum_{i=1}^{m}f_{i}\left(x\right),\\ \text{subject to}\left\{\begin{array}{cc} \frac{f_{i}\left(x\right)-z_{i}^{*}}{z_{i}^{\text{nad}}-z_{i}^{*}}\leq \varepsilon_{i}, & \forall i\in \frac{\left\{1,2,\ldots ,m\right\}}{\left\{s\right\}},\\ x=\left(x_{1},x_{2},\ldots ,x_{n}\right)\in \Omega , \end{array}\right. \end{array}$$

where 0 ≤ *ε*=(*ε*_1_, *ε*_2_,…, *ε*_*s*−1_, *ε*_*s*+1_,…, *ε*_*m*_) ≤ 1 is the upper bound vector, and the index of the main objective is selected from all the objective functions randomly or assigned by the decision-maker. *ρ* is a tiny positive number, *z*^*∗*^=(*z*_1_^*∗*^, *z*_2_^*∗*^,…,*z*_*m*_^*∗*^)^*T*^ and *z*^nad^=(*z*_1_^nad^, *z*_2_^nad^,…,*z*_*m*_^nad^)^*T*^ are the ideal optimal node and ideal worst node, respectively.

The article "MEA-CNDP: A Membrane Evolutionary Algorithm for Solving Biobjective Critical Node Detection Problem" was published in 2021. Journal: Comput Intell Neurosci.

DMOEA-*ε*C proposes the strategy of main objective alternation, which exchanges the main objective function through a specific strategy or periodically and matches the solution with the subproblem again after the main objective function alternation. After a new feasible solution is generated by evolution, DMOEA-*ε*C fits the feasible solution with the subproblem again so that the feasible solution newly generated can be utilized to the maximum extent.

#### 2.3.3. I-MOEA/D and I-DMOEA-*ε*C

MOEA/D and DMOEA-*ε*C perform well on continuous or discrete benchmark problems, but for bi-CNDP, a more special strategy is needed to make them adopt the characteristics of bi-CNDP. Thus, the new mating pool and replacement pool are designed in [31].

In [31], there are four types of strategies for mating pool, including selecting from the neighbors, the whole population, the neighbors and the population, and the external archive population. There are two strategies for the replacement pool, including the local replacement and the global replacement. The experimental results have determined the two algorithms with the best performance, namely, I-MOEA/D and I-DMOEA-*ε*C.

It is worth noting that so far there are few special algorithms to solve bi-CNDP. As the variant of algorithm MOEA/D, I-MOEA/D, and I-DMOEA-*ε*C has shown good results in solving bi-CNDP, inspired by this, this paper aims to explore new better algorithm to solve bi-CNDP; more details are introduced in Section 3.

## 3. The Membrane Evolutionary Algorithm Solving Bi-CNDP

In view of the bi-CNDP introduced above, this section designs and implements the membrane evolutionary algorithm MEA-CNDP solving bi-CNDP. Representation of candidate solutions and related definitions are presented at first. Then, according to the characteristics of bi-CNDP, the membrane evolutionary algorithm framework of MEA-CNDP is designed. Next, some specific strategies are introduced, including population initialization strategy, membrane inherited pool updating, and main objective transforming strategy. Finally, the membrane evolutionary operators, including division, fusion, cytolysis, and selection, are introduced in detail.

### 3.1. Representation and Definition of Candidate Solutions

The initial membrane structure of the MEA-CNDP algorithm is shown in Figure 3. Membrane 0 is the environment membrane (also known as skin membrane) and provides the foundation of the whole membrane population evolving. In the environment membrane, there are the membrane population (membrane 1, 2,…, *N*) for evolution, and the inherited pool (recorded as IP) for each iteration, the external archive membrane (registered as EM) for recording the nondominated solutions. Moreover, all decision variables and upper bound vectors keep only one copy of them in the environment membrane.

The article "MEA-CNDP: A Membrane Evolutionary Algorithm for Solving Biobjective Critical Node Detection Problem" was published in 2021. Journal: Comput Intell Neurosci.

In the process of population evolving, when the individual membrane (membrane *i*) needs to fuse decision variables or upper bound vectors, the decision variables or upper bound vectors are copied into the individual membrane. When an individual membrane is divided, the decision variables and upper bound vectors in it will be dissolved, which means the number of decision variables and upper bound vector in the environment membrane will remain unchanged.

Each evolution only takes place in the membrane population, that is, the division, fusion, cytolysis, and selection operators are only performed in membrane 1, 2,…, *N*. Membrane IP is the current inherited pool, which stores the individual membranes participating in the following evolutionary process. Moreover, the membrane EM is used to record the nondominated solutions in the current membrane population. When a new membrane is generated, the membranes in EM will be updated synchronously. After the evolutionary process is over, the membranes in the EM will output the final solution.

### 3.2. Framework of MEA-CNDP

This section introduces the framework of the proposed MEA-CNDP algorithm. MEA-CNDP performs division, fusion, cytolysis, and selection operators in each evolutionary process and maintains the convergence of the solution by saving and updating the optimal solution. Before each evolutionary process, MEA-CNDP adopts specific strategies to optimize its performance.

The framework of the MEA-CNDP algorithm is shown in Algorithm 2. The parameters of MEA-CNDP are defined as follows:

- *N*: the size of the membrane population, which is the same as the upper bound vector
- *D*: the number of decision variables, which is the same as the number of the nodes in graph
- *T*: the size of neighbors, that is the size of neighbor membrane set of each membrane
- INm: the iteration interval of transforming the main objective function
- DRA_interval: the iteration interval of updating the IP
- *S*: the maximum number of membranes allowed in EM
- *δ*: the probability of selecting from the neighbor membranes when executing the division operator
- Cost_*i*_: the weight of node *i*, which is the cost of deleting node *i* from graph
- Max_Gen_: the maximum number of evolving

Among the above parameters, *T*, INm, DRA_interval, *S*, and *δ* are the parameters of the optimization algorithms, which can be continuously optimized. *N* and Max_Gen_ can be selected by the users. *D* and Cost_*i*_ are definite parameters, which are determined by the dataset.

The article "MEA-CNDP: A Membrane Evolutionary Algorithm for Solving Biobjective Critical Node Detection Problem" was published in 2021. Journal: Comput Intell Neurosci.

In Algorithm 2, MEA-CNDP firstly generates *N* uniformly distributed upper bound vector *ε*^1^, *ε*^2^,…, *ε*^*N*^ by dividing each objective axis with equal spacing Δ.  Figure 4 shows the process of generating upper bound vectors through a 3-objective optimization problem model (*m* = 3), where the equal spacing Δ=1/4 (*q* = 5), 25 upper bound vectors are generated by this way.

MEA-CNDP designs a population initialization strategy; lines 3 and 4 calculate the scores of the decision variables and generate the initial population according to the scores of decision variables, respectively. The initial population generated by the strategy has good characteristics, accelerates the convergence of the population, and maintains diversity. Algorithms 3 and 4 show the details.

Line 5 calculates the neighbor membrane set of each membrane according to Euclidean distance. The value of the upper bound vector of each membrane is used to calculate; thus, *T* neighbor membranes are distributed for each membrane. Line 6 initializes an array of size *N* with all elements values equal to 1, which is used to update the IP.

Line 7 initializes the EM, and the nondominated solutions of all individual membranes in the current membrane population are regarded as the initial object of the EM.

Line 8 initializes the ideal optimal node *Z∗* and ideal worst node *Z*^nad^, which are the minimum and maximum value of each objective function of the present membrane population, respectively. *Z∗* and *Z*^nad^ are updated with the evolutionary process.

The NoF and Cur_Gen_ in lines 9 and 10 mark the main objective and iteration counter, respectively. NoF ∈ {0, 1}, when NoF = 0, the first objective function is selected as the main objective; otherwise, the second objective function is selected. Cur_Gen_ is used to record the number of iterations, and the algorithm ended when Cur_Gen_ meets the maximum iteration number Max_Gen_.

Lines 12–22 are the evolutionary process of each generation in MEA-CNDP. In IP updating (Line 13), the individual membranes in the original IP are removed completely, and Algorithm 5 selects the new individual membranes into IP. In the main objective transforming (Lines 15–16), the upper bound vectors and individual membranes are rematched according to Algorithm 6. The evolution of IP includes membrane division (Algorithm 7) and updated *Z∗*, membrane fusion (Algorithm 8), membrane cytolysis and selection (Algorithm 9), and updated *Z*^nad^.

The article "MEA-CNDP: A Membrane Evolutionary Algorithm for Solving Biobjective Critical Node Detection Problem" was published in 2021. Journal: Comput Intell Neurosci.

Figures 5–8 illustrate the procedure of MEA-CNDP.  Figure 5 shows the membrane structure after one iteration, and the value of Cur_Gen_ will be determined before the next iteration. If the Cur_Gen_ can be divided by DRA_interval_, Algorithm 5 will be executed, and if the Cur_Gen_ can be divided by INm, Algorithm 2 will be executed. Here, we assume that Algorithms 5 and 6 have been executed.  Figure 6 shows the process and results of executing the division operator. In one evolution, according to Algorithm 7, membranes *m*_*j*_ and *m*_3_ are selected to perform the division operation, and membrane *o* is the generated offspring membrane.  Figure 7 shows the process and results of performing the fusion operator. According to Algorithm 8, the upper bound vector of membrane *o* and the substances in the neighbor membrane of membrane *o* are updated.  Figure 8 shows the process and results of performing the cytolysis and selection operator. According to Algorithm 9, the membrane *o* interacts with the membrane in the external archive membrane EM, dissolves the bad membrane, and selects the retained membrane.

MEA designs evolutionary strategy according to the information exchange between membranes. According to the life activities of membrane and the information exchange mechanism between membranes, MEA generates its own unique division, fusion, dissolution, and selection operators. MEA uses membrane heuristic information and parallel optimization to realize individual evolution and solve problems. In particular, MEA-CNDP takes into account the characteristics of the bi-CNDP and introduces new strategies such as population initialization and new evolutionary operators, thereby establishing a new framework to solve bi-CNDP.

### 3.3. The Initialization Strategy

The pro and cons of the initial population significantly affect the bi-CNDP, especially for the models similar to large-scale MOPs. Thus, MEA-CNDP introduces a population initialization strategy, which includes two parts: evaluating the scores of decision variables and generating the initial population. Through this strategy, not only can the quality of the initial population be improved but it can also provide evidence for deciding whether to retain or eliminate evolutionary genes.

The process of calculating the scores of decision variables can be seen in Algorithm 3, the coding method is used in [37], and some improvement is executed according to the characteristic of bi-CNDP. Firstly, since the decision variable of bi-CNDP is a binary value (if the node is deleted, the value of the corresponding decision variable will be set to 1; otherwise, it is 0), Algorithm 3 simplifies the coding process, adopts binary coding directly, and omits the real vector coding of the solution. Next, in bi-CNDP, the degree of a node is taken into account. Nodes with degree 1 are not included in the score calculating of the decision variables (in fact, their scores have been assigned to Max_Double). Deleting nodes with degree 1 in the graph has little effect on the pairwise connectivity of the graph. Especially in the large-scale graph, the effect is almost negligible. On the contrary, it will increase the impact on “minimize deleting cost.” Finally, because the nodes in bi-CNDP have weights related to the cost of deleting themselves, the final calculation results will be determined by the nondominated front number and the cost of deleting the corresponding node together, which can more accurately assess the importance of each decision variable.

The article "MEA-CNDP: A Membrane Evolutionary Algorithm for Solving Biobjective Critical Node Detection Problem" was published in 2021. Journal: Comput Intell Neurosci.

Algorithm 4 shows the process of generating the initial population. Each individual membrane is generated by adding decision variables to the empty membrane, and the selected decision variables are determined by comparing their scores. The size of each membrane is set as rand() × *D*, which is seen as a random parameter. The decision variables with smaller score values are more likely to be selected because the smaller score values often mean better nondominated solutions.

### 3.4. Membrane Inherited Pool Updating and Main Objective Transforming

Different individuals in the membrane population have different upper bound vectors and subproblems, which means that the calculation difficulty is also different. Therefore, it is reasonable to assign different amounts of computational effort to different individuals according to the utility value in each generation of evolution. Algorithm 5 updates the IP through fixed iteration interval, and in each evolutionary process, only the individual membranes in IP participate in the evolution, which ensures the efficiency of the MEA-CNDP algorithm.

Algorithm 5 calculates the utility value of each individual membrane in Lines 6–9. Every time the IP is updated, all individual membranes in the original IP are removed. Line 14 selects several individual membranes to enter the IP through binary tournament selection, which means that the individual membrane with better utility value will be more likely to enter the IP. This process is repeated (*N*/5 − *m* − 1) times to select adequate individual membranes, and these individual membranes in the IP participate in the evolutionary process until the IP is updated next time. The details of parameter selection can be seen in [35].

The article "MEA-CNDP: A Membrane Evolutionary Algorithm for Solving Biobjective Critical Node Detection Problem" was published in 2021. Journal: Comput Intell Neurosci.

Since transforming the main objective is adopted, the main objective function will convert with a fixed iteration interval. Among the current membrane population, the individual membranes that perform well to the original main objective function may not perform well to the current main objective function; thus, it is necessary to rematch the membrane and the subproblem.

Algorithm 6 matches the individual membrane with the smallest distance from a certain subproblem (in fact, different upper bound vector represents different subproblem) in *N* individual membranes to the subproblem. Line 8 defined the formula of calculating the distance. This matching strategy is implemented after transforming the main objective function, which means each upper bound vector is combined with the fittest subproblem throughout. By implementing this strategy, the excellent individuals will not be eliminated because of a single evaluation standard; thus, the diversity of the membrane population is maintained.

### 3.5. Evolutionary Operator

#### 3.5.1. Division Operator

In the evolutionary process, the division operator is used to generate new individual membranes based on the existing heuristic information to ensure that the membrane population always evolves in a better direction. Algorithm 7 shows the implementation process of the division operator.

One of the parent membranes used to perform division operator comes from the EM, and another comes from the whole membrane population or the neighbor membranes of the current membrane depending on probability. In the process of division operator, the decision variables shared by the two parental membranes are retained firstly, and then the decision variables unique to the two parental membranes are removed or retained by equal probability. In removing or keeping decision variables, the selection is made based on the score of the decision variable, the decision variable with a smaller score will be retained, and the decision variable with a larger score will be removed. Finally, to avoid the membrane population falling into the local optimum, the decision variables are released from the membrane to the environment or copied from the environment to the membrane with equal probability. Similarly, the decision variables with a larger score in the individual membrane will be released, while the decision variables with a smaller score in the environment will be copied into the individual membrane.

#### 3.5.2. Fusion Operator

When the division operator generates a new individual membrane, it may not perform well for the subproblem corresponding to the upper bound vector in its membrane, but performs well for the subproblem corresponding to another upper bound vector. So, Algorithm 8 fuses the newly generated individual membrane with the other upper bound vector, and the neighbor membrane will also be updated.

The article "MEA-CNDP: A Membrane Evolutionary Algorithm for Solving Biobjective Critical Node Detection Problem" was published in 2021. Journal: Comput Intell Neurosci.

Algorithm 8 contains two parts. Firstly, the newly generated individual membrane is fused with another upper bound vector suitable itself, to avoid the waste of the newly generated excellent individual membrane because it does not adapt to its own upper bound vector. Lines 1–6 define the steps to search the upper bound vector corresponding to the newly generated individual membrane, which is conducive to the convergence of the membrane population. Then, according to the objective function value of the newly generated individual membrane, the neighbor membranes are updated, the nondominated individual membrane is retained, and the dominated solution is removed.

#### 3.5.3. Cytolysis and Selection Operator

The selection and cytolysis operator updates the EM by calculating the dominant relationship between the newly generated individual membrane and the individual membrane in the EM. All the individual membranes dominated by the newly generated individual membrane in the external archive membrane will be dissolved. If no individual membrane dominates the newly generated individual membrane in the EM, the newly generated individual membrane will be added to the EM. Algorithm 9 shows the selection and cytolysis operator in detail.

These four evolutionary operators occurred during the evolution of the entire membrane population. The division operator produces better individual membrane, the fusion operator matches the individual membrane with the appropriate upper bound vector, and the selection and cytolysis operator guarantees the quality of the EM. The execution of different operators promotes the exchange of information between membranes and makes the entire membrane population continue to evolve.

In general, MEA-CNDP is a new MEA framework for solving bi-CNDP. The main features of the MEA-CNDP algorithm are as follows: (1) since each membrane represents an individual, the entire solving process can be realized entirely through membrane evolving. (2) The evolutionary process includes not only the evolution of the objects in the membrane but also the evolution of the membrane structure, so that excellent individuals can always be maintained. (3) Since the substance stored in the membrane can be any object, the complexity of encoding different evolutionary objects is avoided. (4) The evolutionary strategy guarantees the maximum theoretical parallelism of the evolutionary process and greatly improves the efficiency of the algorithm. To verify the effectiveness and efficiency of MEA-CNDP, based on four different types and sixteen different sizes of CNDP instances, this paper designs relative comparative experiments of the MEA-CNDP algorithm and some other algorithms, and the relevant results will be introduced in Section 4.

The article "MEA-CNDP: A Membrane Evolutionary Algorithm for Solving Biobjective Critical Node Detection Problem" was published in 2021. Journal: Comput Intell Neurosci.

## 4. Numerical Experiments

This section is devoted to design related experiments to verify the effectiveness of the proposed MEA-CNDP algorithm and compare it with other existing algorithms on bi-CNDP. Specifically, four different types of benchmark problems and datasets of CNDP are outlined firstly. As each type of problem possesses four different sizes of datasets, 16 benchmark instances, the parameter characteristics of all instances are introduced as well. To compare the performance of different algorithms objectively, the experimental performance measures are given secondly. Then, the parameters of all the algorithms involved are provided, as well as the experimental environment. Finally, the experimental results of the MEA-CNDP and other algorithms are shown, and further analysis of the results proves the effectiveness of the MEA-CNDP.

### 4.1. The Benchmark Problems and Dataset of CNDP

Since there are no specific datasets for the biobjective critical node detection problem, all of the instances of this paper are composed of the graphs of several complex networks [27]. These graphs are usually studied as single-objective critical node detection problem, and many effective results have been obtained. The datasets contain 16 undirected unweighted graphs, all of which are created by complex network generator algorithms. However, few studied deal with them as MOPs, which are also the motivations and inspirations of this paper.

The datasets are divided into four types. Barabasi–Albert (BA) graphs start from a small number of nodes, enriches the network with the increase of nodes and edges over time, and finally forms a scale-free complex network graph, which is proved to be the easiest to process in related data sets. Watts–Strogatz (WS) graphs simulate a small world with a more intensive structure, that is, the diameter of the graph is small, and most nodes can access each other in relatively few hops, which is the most challenging. Edros–Renyi (ER) graphs are random, and every pair of vertices in the graph are randomly connected to form edges according to the probability, to form a completely random graph. Forest-Fire (FF) graphs simulate the model of fire spreading in a forest, different from BA, FF reproduces the heavy tailed distribution, and the network diameter decreases with time. It is worth noting that although these digitized instances cannot be reproduced in real networks, the real complex networks often show the combination of features in these datasets.

The article "MEA-CNDP: A Membrane Evolutionary Algorithm for Solving Biobjective Critical Node Detection Problem" was published in 2021. Journal: Comput Intell Neurosci.

For these critical node detection problems, it is vital to take into account the number of deleted nodes and the cost of deleting nodes at the same time. Therefore, it is worthy to consider them from the perspective of MOPs. MEA has been proved to have its own unique advantages in solving combinatorial optimization problems [14–16]. Besides, the proposed MEA algorithm in this paper takes into account the sparsity and large-scale characteristics of the above application data sets, so it shows excellent performance. The experimental results are detailed in Section 4.4.

In order to characterize the graph structure of the above datasets accurately, some related quantities are shown in Table 1. *n* is the number of nodes, *m* is the number of edges, 〈*d*〉 represents the average degree of nodes, which can be formulated as 〈*d*〉=2 · *m*/*n*, and nAP represents the number of articulation nodes. CC represents the value of the clustering coefficient, *D* represents the average shortest path length [28], |*D*_1_| represents the number of nodes having degree 1, and *N*(|*D*_1_|) represents the number of nodes whose neighboring nodes having degree 1 [36]. Among these characteristics, consider the number of articulation nodes nAP because the graph with larger nAP is easier to fragment. The clustering coefficient CC can describe the clustering tendency of nodes. The average shortest path length *D* represents the average distance between two randomly selected nodes in the graph.

Since these networks are not weighted in the original network, new benchmark instances are created by assigning a weight value to each node of each network, and the weight of each node is regarded as the cost of removing the node. The weight generation method comes from [31] and can be described as follows:

1. Assign weight to nodes randomly, for example, cost(*v*) ∈ [0.2, 3], ∀*v* ∈ *V*
2. Assign weight to nodes according to the degree, for example, cost(*v*)=log(*d*_*v*_)+0.5, ∀*v* ∈ *V*, where *d*_*v*_ represents the degree of the node

### 4.2. Performance Measures

In this paper, the inverted generational distance (IGD) [37, 38] and the hypervolume (HV) [39, 40] are chosen as performance measures.

#### 4.2.1. IGD

IGD can provide combined information on the convergence and diversity of the known solution. Therefore, it is widely used to evaluate the approximate solution set of MOPs.

Let *P*^*∗*^ denote a subset of pareto-optimal solutions uniformly distributed along with the true PF and *P* be an approximation set obtained by multiobjective optimization algorithms. The IGD measures the average distance from each point in *P*^*∗*^ to its nearest point in P regarding the objective space. It is calculated as

(6) $$\begin{array}{c} \text{IGD}\left(P^{*},P\right)=\frac{\sum_{x\in P^{*}}d\left(x,P\right),}{\left|P^{*}\right|} \end{array}$$

where *d*(*x*, *P*) represents the Euclidean distance from *x* to its nearest neighbor in *P*. Generally, a smaller IGD value indicates a better convergence and diversity of *P*. In MEA-CNDP, for calculating IGD, *N* nondominated solutions are selected from the external membrane using the crowding distance approach [41]. *P*^*∗*^ is chosen from the combination of all the solutions obtained by the experiments over 20 independent runs.

The article "MEA-CNDP: A Membrane Evolutionary Algorithm for Solving Biobjective Critical Node Detection Problem" was published in 2021. Journal: Comput Intell Neurosci.

#### 4.2.2. HV

HV is used to calculate the volume covered by the obtained dominant individual in the objective space, especially when the true PF of the MOPs in the application are unknown. It is calculated as

(7) $$\begin{array}{c} \text{HV}=\text{volume}\left(\overset{n_{\text{PF}}}{\underset{i=1}{\cup }}v_{i}\right), \end{array}$$

where *n*_PF_ is the number of nondominated individuals in the approximation solution sets. For every individual *i* in the nondominated solution set, *v*_*i*_ is the hypervolume of reference point *ω* and individual member *i*. In MEA-CNDP, for calculating HV, the reference point *ω* is set as 1.1 times the nadir point in *P*^*∗*^ for each instance.

### 4.3. Experimental Environment and Parameter Setting

So far, algorithms I-MOEA/D and I-MOEA/D-*ε*C have shown the best results in solving bi-CNDP; therefore, this paper analyzes and compares the proposed MEA-CNDP algorithm with these two algorithms. To be fair, the relevant parameters are set as follows: Algorithms I-MOEA/D and I-MOEA/D-*ε*C use the same parameters and use binary vectors to encode the feasible solution. For algorithms I-MOEA/D, I-MOEA/D-*ε*C, and MEA-CNDP, the population size *N* is set as 300, 400, 500, and 600 for each instance when the number of nodes is *n* ≤ 500, 500 < *n* ≤ 1000, 1000 < *n* ≤ 2500, and 2500 < *n* ≤ 5000. For the external population of algorithms I-MOEA/D and I-MOEA/D-*ε*C, the external membrane of algorithm MEA-CNDP, the size *S* is set as *S*=⌊1.5 · *N*⌋, where ⌊·⌋ returns the nearest integer in the negative infinity direction.

For algorithms I-MOEA/D and I-MOEA/D-*ε*C, the parameterized uniform crossover [42] and random mutation [22] are adopted to generating new candidate solutions. Besides, the control parameters of the related generation operation are the same as those in [22], that is, the biased probability of crossover is set as 0.65, and the random mutation probability of each decision variable of the solution is set as 0.03.

The article "MEA-CNDP: A Membrane Evolutionary Algorithm for Solving Biobjective Critical Node Detection Problem" was published in 2021. Journal: Comput Intell Neurosci.

For algorithms I-MOEA/D, I-MOEA/D-*ε*C and MEA-CNDP, the size of the neighborhood is set as ⌊0.1 · *N*⌋, the probability of selecting an individual from the neighborhood is set as 0.9. For algorithms I-MOEA/D and I-MOEA/D-*ε*C, the maximal number of replacement is set as ⌊0.01 · *N*⌋. The maximum number of iterations *I* is set as 2500, 4000, 6000, and 7500 when the number of nodes is *n* ≤ 500, 500 < *n* ≤ 1000, 1000 < *n* ≤ 2500, and 2500 < *n* ≤ 5000. For algorithms I-MOEA/D-*ε*C and MEA-CNDP, the iteration interval of transforming the main objective function is set as ⌊20%·*I*⌋. When the number of iterations reaches the maximum, all algorithms end.

All comparison algorithms are run on a personal computer with a 2.20 GHz CPU and 8 GB RAM. Each algorithm runs independently 20 times to obtain statistical results.

### 4.4. Experimental Results and Analysis

As mentioned above, the comparative experiments are carried out in three algorithms (i.e., I-MOEA/D, I-MOEA/D-*ε*C and MEA-CNDP). Considering I-MOEA/D, I-MOEA/D-*ε*C and their variants, only the best results among their various variants are considered in the following experiments, that is, in the mating pool selection strategy, the “-NP-EP” method is adopted, and the “-G” method is adopted in the replacement pool strategy. All of the experimental results of I-MOEA/D and I-MOEA/D-*ε*C are from [31]. Tables 2–5 exhibit the total comparative experimental results of the three algorithms. The values in Tables 2 and 3 are the average IGD on all test instances with random weights and logarithmic weights, respectively. The values in Tables 4 and 5 are the average HV on all test instances with random weights and logarithmic weights, respectively. For each indicator, the bold data in each table are the best mean metric values of each instance. Noteworthy is that, for fair comparison, the same parameters in the three algorithms are given the same values. As for the specific parameter in MEA-CNDP algorithm, the experiments to detect the influence of parameters on the experimental results are designed and implemented, and therefore, the excellent parameters are selected. The experimental results in the tables are the results of selecting better parameters.

Tables 2 and 3 show the results of the IGD metric values on all test instances with random weights and logarithmic weights. As shown in Table 2, in 16 test instances with random weights, the MEA-CNDP algorithm performs better than other algorithms in 11 instances. Further analysis can find that, in all instances of BA and FF of four different sizes, the MEA-CNDP algorithm also has significant advantages over other algorithms. Moreover, the MEA-CNDP algorithm shows poor results in the WS instance. In ER instance, the MEA-CNDP algorithm and I-MOEA/D-*ε*C algorithm show competitive performance. The experimental results in Table 3 show that, in 16 test instances with logarithmic weights, the MEA-CNDP algorithm performs better than other algorithms in 10 instances. Specifically, in 16 instances, the MEA-CNDP algorithm shows absolute advantage in BA and FF instances with all sizes of graphs and shows slightly worse results in WS and ER instances.

The article "MEA-CNDP: A Membrane Evolutionary Algorithm for Solving Biobjective Critical Node Detection Problem" was published in 2021. Journal: Comput Intell Neurosci.

Tables 4 and 5 show the results of the HV metric values on all test instances with random weights and logarithmic weights. Different from the experimental results of the IGD metric, it is evident that the performance of the MEA-CNDP algorithm in the HV metric is far better than the other algorithms. Specifically, the MEA-CNDP algorithm achieves the best solution on all sizes of 16 instances with random weights and achieves the best on 15 out of 16 instances with logarithmic weights, proving that the MEA-CNDP algorithm possesses good convergence and population diversity.

It can be seen from the results of the above comparative experiments that, MEA-CNDP algorithm has good performance for most of the instances, except for the WS and ER instances.

To better measure the performance of MEA-CNDP more accurately, further experiments of I-MOEA/D-*ε*C and MEA-CNDP algorithms are carried out. Figures 9 and 10 exhibit the degree of improvement of the MEA-CNDP algorithm relative to the I-MOEA/D-*ε*C algorithm. In Figure 9, PIR_IGD_ is calculated by formula (8), and IGD(*A*) represents the IGD metric of algorithm *A*. PIR_IGD_ represents the relative change rate of the IGD metric of the algorithms MEA-CNDP and MOEA/D-*ε*C as the number of decision variables increases. The smaller the IGD, the better the solution. So, MEA-CNDP shows worse results than I-MOEA/D-*ε*C in small-scale instances of WS and ER. However, with the increase of the number of decision variables, the MEA-CNDP algorithm shows better results.

(8) $$\begin{array}{c} {\text{PIR}}_{\mathrm{IGD}}=\frac{\text{IGD}\left(\text{I}-\text{DMOEA}-\varepsilon \text{C}\right)-\text{IGD}\left(\text{MEA}-\text{CNDP}\right)}{\text{IGD}\left(\text{I}-\text{DMOEA}-\varepsilon \text{C}\right)}. \end{array}$$

In Figure 10, PIR_HV_ is calculated by formula (9), and HV(*A*) represents the HV metric of algorithm *A*. PIR_HV_ represents the relative change rate of the HV metric. The larger the HV, the better the solution, which means that the MEA-CNDP algorithm is always better than the I-MOEA/D-*ε*C algorithm in HV metric, and this advantage becomes more obvious as the number of decision variables increases. Thus, it can be seen that the MEA-CNDP algorithm possesses better adaptability for large-scale MOPs.

(9) $$\begin{array}{c} {\text{PIR}}_{\mathrm{HV}}=\frac{\text{HV}\left(\text{MEA}-\text{CNDP}\right)-\text{HV}\left(\text{I}-\text{DMOEA}-\varepsilon \text{C}\right)}{\text{HV}\left(\text{I}-\text{DMOEA}-\varepsilon \text{C}\right)}. \end{array}$$

In addition, some potential knowledge can be derived from the initialization strategy of the MEA-CNDP. Algorithms 3 and 4 introduce the evaluation method of decision variables and the initial population generation strategy, respectively. Among them, for evaluating the score value of decision variables, Algorithm 3 eliminates the consideration of nodes with degree 1 and considers those with a degree greater than 1 because deleting the nodes with degree 1 in the graph will only have a small impact on calculating the pairwise connectivity of the residual graph. It can be seen from Table 1 that there are no nodes with degree 1 in WS instances and only a few nodes with degree 1 in ER instances; in other words, WS and ER instances are relatively denser graphs. Furthermore, Algorithms 3 and 4 consider the ratio of the nondominated front number to the cost of deleting nodes as the scores of decision variables, which also shows that the MEA-CNDP algorithm is more suitable for sparse graphs.

The article "MEA-CNDP: A Membrane Evolutionary Algorithm for Solving Biobjective Critical Node Detection Problem" was published in 2021. Journal: Comput Intell Neurosci.

An excellent initial population will have a significant impact on the subsequent solution space search. As can be seen, the I-MOEA/D-*ε*C algorithm uses the random initialization strategy; in contrast, MEA-CNDP designs the above specific initialization strategy.  Figure 11 shows the population generated by the initialization strategy of MEA-CNDP and random initialization strategy in the objective space, and each population contains 50 solutions for the four types of instances of 500 decision variables with random weights, where *f*_1_ and *f*_2_ are two objective function values. Not difficult to see from Figure 11, the random population initialization strategy often has poor convergence and population diversity, so that it is easy to cause the subsequent search to fall into the local optimum, thereby deteriorating the entire algorithm process. In contrast, the population initialization strategy of the MEA-CNDP algorithm considers the characteristics of each decision variable itself. It performs the necessary screening of the solution when the population is initialized, so that the entire initial population has a higher quality, which is undoubtedly beneficial to produce a better solution. This also shows that our strategy has greater advantages when facing large-scale sparse graphs such as BA and FF instances.

The article "MEA-CNDP: A Membrane Evolutionary Algorithm for Solving Biobjective Critical Node Detection Problem" was published in 2021. Journal: Comput Intell Neurosci.

## 5. Conclusion and Future Work

As a classical problem in combinatorial optimization, CNDP is often studied as a single-objective optimization problem. However, this kind of research method has some limitations and cannot cover all the problems. In addition, as a kind of new evolutionary algorithm, MEA has its unique advantages in solving such combinatorial optimization problems with graph properties. Therefore, this paper is devoted to research a membrane evolution algorithm to solve the problem of bi-CNDP (MEA-CNDP). In MEA-CNDP, a population initialization method based on decision variable evaluation is proposed. Then, some measures to enhance the efficiency of the MEA-CNDP algorithm are presented, including the main objective function transforming, membrane and subproblem matching strategies. Finally, according to the algorithm framework of MEA-CNDP, we design and implement the correlation division, fusion, cytolysis, and selection operators. To verify the effectiveness of MEA-CNDP, the comparative experiments are designed. The experimental results show that MEA-CNDP has good performance in solving bi-CNDP.

For future work, there are two potential research directions. At first, the population initialization strategy is worth further consideration, a more accurate method to calculate the score of the decision variable can be designed, and updating the score of the decision variable in the evolutionary process is considerable as well. Another interesting research direction is considering some local search strategies in the design of evolutionary operators, which can further enhance the quality of solutions.

## Figures and Tables

**Figure 1:** The schematic diagram of the nested structure of MA.

**Figure 2:** The schematic diagram of the division and fusion operator. (a) Division operator. (b) Fusion operator.

**Figure 3:** The initial membrane structure of the MEA-CNDP algorithm.

**Figure 4:** The process of generating uniformly distributed upper bound vector.

**Figure 5:** The membrane structure before the beginning of a certain evolution.

**Figure 6:** The membrane structure of performing the division operator.

**Figure 7:** The membrane structure of performing the fusion operator.

**Figure 8:** The membrane structure of performing the cytolysis and selection operator.

**Figure 9:** The PIR changes with the increase in the number of decision variables of the IGD metric of WS and ER instances on random and logarithmic weights. (a) WS instance. (b) ER instance.

**Figure 10:** The PIR changes with the increase in the number of decision variables of the HV metric of WS and ER instances on random and logarithmic weights. (a) WS instance. (b) ER instance.

The article "MEA-CNDP: A Membrane Evolutionary Algorithm for Solving Biobjective Critical Node Detection Problem" was published in 2021. Journal: Comput Intell Neurosci.

**Figure 11:** Initial population generated by the initialization strategy of MEA-CNDP and a randomly generated population in objective space. (a) BA instance. (b) WS instance. (c) ER instance. (d) FF instance.

**Algorithm 1:** Framework of MEA.

**Algorithm 2:** Framework of MEA-CNDP. The MEA solving bi-CNDP.

**Algorithm 3:** Score_Assignment. Calculate the scores of decision variables.

**Algorithm 4:** Initialize_Population. Generate the initial membrane population.

**Algorithm 5:** UpdateIP. Update the membrane inherited pool.

**Algorithm 6:** Membrane-to-subproblem matching.

**Algorithm 7:** Division.

**Algorithm 8:** Fusion.

**Algorithm 9:** Cytolysis and Selection.

**Table 1:** Some related quantities of the sixteen benchmark instances.

Instance	*n*	*m*	<*d*>	*n*AP	CC	D	|*D*_1_|	*N*(|*D*_1_|)
BA500	500	499	1.996	164	0	5.663	336	149
BA1000	1000	999	1.998	324	0	6.045	676	290
BA2500	2500	2499	1.999	825	0	6.901	1675	729
BA5000	5000	4999	1.999	1672	0	8.38	3328	1475
WS250	250	1246	9.968	0	0.473	3.327	0	0
WS500	500	1496	5.984	0	0.42	5.304	0	0
WS1000	1000	4996	9.992	0	0.483	4.444	0	0
WS1500	1500	4498	5.997	0	0.48	7.554	0	0
ER235	235	350	2.979	48	0.006	5.339	39	37
ER466	466	700	3.004	84	0.002	5.974	69	64
ER941	941	1400	2.976	177	0.005	6.559	147	139
ER2344	2344	3500	2.986	419	0.001	7.516	396	354
FF250	250	514	4.112	83	0.276	4.816	57	50
FF500	500	828	3.312	195	0.247	6.026	160	136
FF1000	1000	1817	3.634	362	0.216	6.173	280	236
FF2000	2000	3413	3.413	725	0.245	7.587	552	477

**Table 2:** The experimental results of IGD of MEA-CNDP and other algorithms on random weights instance.

Instance	I-MOEA/D	I-DMOEA-*ε*C	MEA-CNDP
BA500	3.19*E* − 03	1.74*E* − 04	**1.66 ** *E* − **04**
BA1000	1.57*E* − 02	5.76*E* − 04	**2.49 ** *E* − **04**
BA2500	4.74*E* − 04	4.64*E* − 04	**9.95 ** *E* − **05**
BA5000	7.57*E* − 03	7.34*E* − 04	**4.60 ** *E* − **04**
WS250	2.23*E* − 02	**9.36 ** *E* − **04**	5.85*E* − 03
WS500	1.50*E* − 02	**6.23 ** *E* − **04**	3.84*E* − 03
WS1000	1.65*E* − 02	**1.40 ** *E* − **03**	6.14*E* − 03
WS1500	4.89*E* − 02	4.27*E* − 03	**4.14 ** *E* − **03**
ER235	3.52*E* − 02	**2.64 ** *E* − **04**	8.04*E* − 04
ER466	8.79*E* − 03	**8.64 ** *E* − **04**	2.46*E* − 03
ER941	2.70*E* − 02	4.62*E* − 03	**2.20 ** *E* − **03**
ER2344	2.28*E* − 02	6.99*E* − 03	**1.99 ** *E* − **03**
FF250	5.20*E* − 02	9.84*E* − 04	**1.18 ** *E* − **04**
FF500	3.75*E* − 02	2.73*E* − 03	**1.45 ** *E* − **03**
FF1000	2.28*E* − 02	1.33*E* − 03	**1.14 ** *E* − **03**
FF2000	2.58*E* − 02	2.81*E* − 03	**9.36 ** *E* − **04**

**Table 3:** The experimental results of IGD of MEA-CNDP and other algorithms on logarithmic weights instance.

Instance	I-MOEA/D	I-DMOEA-*ε*C	MEA-CNDP
BA500	3.41*E* − 02	2.13*E* − 04	**1.33 ** *E* − **04**
BA1000	6.16*E* − 03	4.21*E* − 04	**3.03 ** *E* − **04**
BA2500	2.77*E* − 02	6.19*E* − 04	**2.34 ** *E* − **04**
BA5000	6.05*E* − 03	5.48*E* − 04	**3.33 ** *E* − **04**
WS250	2.28*E* − 02	**4.82 ** *E* − **04**	8.49*E* − 03
WS500	7.86*E* − 03	**6.16 ** *E* − **03**	1.53*E* − 02
WS1000	9.84*E* − 03	**8.15 ** *E* − **04**	1.02*E* − 03
WS1500	7.15*E* − 03	6.42*E* − 04	**6.33 ** *E* − **04**
ER235	2.19*E* − 02	**5.92 ** *E* − **04**	1.80*E* − 03
ER466	1.42*E* − 02	**2.62 ** *E* − **03**	4.40*E* − 03
ER941	2.35*E* − 03	**2.52 ** *E* − **03**	3.94*E* − 03
ER2344	7.54*E* − 03	6.17*E* − 04	**4.03 ** *E* − **04**
FF250	5.19*E* − 02	4.10*E* − 03	**2.07 ** *E* − **03**
FF500	1.30*E* − 02	9.19*E* − 04	**8.02 ** *E* − **04**
FF1000	9.05*E* − 02	6.81*E* − 03	**6.26 ** *E* − **03**
FF2000	3.24*E* − 02	4.46*E* − 03	**3.78 ** *E* − **03**

The article "MEA-CNDP: A Membrane Evolutionary Algorithm for Solving Biobjective Critical Node Detection Problem" was published in 2021. Journal: Comput Intell Neurosci.

**Table 4:** The experimental results of HV of MEA-CNDP and other algorithms on random weights instance.

Instance	I-MOEA/D	I-DMOEA-*ε*C	MEA-CNDP
BA500	9.15*E* − 03	6.81*E* − 02	**3.52 ** *E* − **01**
BA1000	8.81*E* − 05	4.33*E* − 04	**3.24 ** *E* − **03**
BA2500	8.87*E* − 06	4.55*E* − 05	**1.09 ** *E* − **04**
BA5000	6.48*E* − 05	7.56*E* − 05	**1.20 ** *E* − **04**
WS250	3.44*E* − 01	4.04*E* − 01	**7.49 ** *E* − **01**
WS500	2.89*E* − 01	3.57*E* − 01	**5.56 ** *E* − **01**
WS1000	3.95*E* − 02	3.17*E* − 02	**8.20 ** *E* − **02**
WS1500	6.61*E* − 02	7.67*E* − 02	**4.10 ** *E* − **01**
ER235	2.98*E* − 01	4.23*E* − 01	**5.81 ** *E* − **01**
ER466	1.16*E* − 01	3.45*E* − 01	**5.23 ** *E* − **01**
ER941	2.48*E* − 02	4.89*E* − 02	**9.14 ** *E* − **02**
ER2344	5.41*E* − 05	2.25*E* − 04	**1.15 ** *E* − **03**
FF250	1.37*E* − 01	4.22*E* − 01	**7.20 ** *E* − **01**
FF500	7.11*E* − 02	1.19*E* − 01	**5.32 ** *E* − **01**
FF1000	4.96*E* − 03	1.72*E* − 02	**5.22 ** *E* − **02**
FF2000	3.86*E* − 04	5.67*E* − 04	**1.20 ** *E* − **03**

**Table 5:** The experimental results of HV of MEA-CNDP and other algorithms on logarithmic weights instance.

Instance	I-MOEA/D	I-DMOEA-*ε*C	MEA-CNDP
BA500	5.25*E* − 02	1.89*E* − 01	**9.20 ** *E* − **01**
BA1000	1.39*E* − 04	5.95*E* − 04	**1.20 ** *E* − **03**
BA2500	5.59*E* − 05	4.54*E* − 05	**3.66 ** *E* − **04**
BA5000	4.99*E* − 05	6.58*E* − 05	**1.21 ** *E* − **04**
WS250	3.41*E* − 01	**4.49 ** *E* − **01**	4.10*E* − 01
WS500	1.58*E* − 01	2.77*E* − 01	**9.10 ** *E* − **01**
WS1000	1.75*E* − 01	6.51*E* − 02	**2.53 ** *E* − **01**
WS1500	2.54*E* − 02	7.73*E* − 02	**4.20 ** *E* − **01**
ER235	3.05*E* − 01	5.78*E* − 01	**1.09 ** *E* + **00**
ER466	1.24*E* − 01	2.16*E* − 01	**8.40 ** *E* − **01**
ER941	9.53*E* − 03	1.68*E* − 02	**9.80 ** *E* − **02**
ER2344	6.47*E* − 04	6.01*E* − 04	**3.97 ** *E* − **03**
FF250	2.68*E* − 01	5.62*E* − 01	**1.12 ** *E* + **00**
FF500	3.88*E* − 02	6.09*E* − 02	**1.70 ** *E* − **01**
FF1000	3.77*E* − 03	7.74*E* − 03	**1.50 ** *E* − **02**
FF2000	4.22*E* − 03	9.89*E* − 03	**5.17 ** *E* − **02**

The article "MEA-CNDP: A Membrane Evolutionary Algorithm for Solving Biobjective Critical Node Detection Problem" was published in 2021. Journal: Comput Intell Neurosci.

## Data Availability

All the original experimental data in this article are from http://individual.utoronto.ca/mventresca/cnd.html.
